The article "Mate Analysis of Hepatocellular Carcinoma Immune Subtypes and Their Functional Effects Based on Fuzzy Logic and Evolutionary Algorithms" was retracted in 2023. Reasons: suspected computer-generated content; unreliable results or conclusions; concerns about the data; concerns about the results or conclusions.

# Mate Analysis of Hepatocellular Carcinoma Immune Subtypes and Their Functional Effects Based on Fuzzy Logic and Evolutionary Algorithms

**DOI:** 10.1155/2022/5787981

**Published:** 2022-05-05

**Authors:** Qingge Chen, Chaoyi Liu, Yujia Huo

**Affiliations:** Huanghe Science & Technology University, Zhengzhou, Henan 450063, China

## Abstract

Functional analysis of immune subtypes in hepatocellular carcinoma has attracted much attention due to its advantages in solving some optimization problems. At present, the research on the immune subtype of hepatocellular carcinoma is still in its infancy, and the high stability of its system still has problems. Based on fuzzy logic and evolutionary algorithms, this paper constructs a Mate analysis of the optimization problem of immune subtypes and dynamic optimization problems of hepatocellular carcinoma. The model conducts in-depth analysis and research on the biological immune subtype system, solving the problems of reliable information processing and body defense. Tested with existing test functions, very competitive results were achieved. The simulation results show that the improved algorithm based on data statistics has global search ability, the solution accuracy reaches 0.931, and the stability reaches 88.1%.

## 1. Introduction

For the Mate optimization of fuzzy evolutionary algorithm, the previous research was applied to the process control of a second-order object, the MATLAB simulation test was carried out, and good results were obtained. The optimization effect has been further tested, and the results show that it can be used to optimize the Mate parameters of the Mate controller to improve its control performance and improve the control effect, safety, and economic benefits [1]. Comparing with the previous algorithms, the experiment finally shows the ubiquity, superiority, and practicability of the fuzzy evolutionary algorithm, which can be applied in many algorithm optimizations. In addition to the properties mentioned above, description logic can use subconcept (parent concept) relationships (containment relationships) to structure the concept hierarchy in a given term set, so term sets are often constructed as a hierarchical tree of containment relationships. Such a hierarchical structure provides great convenience for establishing connections between different concepts. In addition, such a mechanism can also improve the efficiency of reasoning services to a certain extent [2–4].

However, the immune subtype system itself is more complex, so there are relatively few studies on artificial immune subtype system models. Although the existing research results show the great potential of artificial immune subtype algorithm in solving some practical problems and the advantages in solving some optimization problems, the current research on artificial immune subtype system algorithms is still in its infancy. Its broad application prospects are still waiting for more detailed development [5]. In order to improve the search speed of the algorithm, the gradient-like information is extracted from the redundant information carried by the cloned individuals, which expands the application range of commonly used gradient information extraction methods such as traditional Jacobian vector and tangent vector, improves the search performance of the algorithm, and strengthens the interaction between individuals in subgroups and between subgroups; deleting to cope with the dynamic characteristics of dynamic optimization of periodic and nonperiodic changes, the memory mechanism of immune subtypes of hepatocellular carcinoma was deeply studied; and according to the different life cycles of memory hepatocytes, the proposed long-term-short-term memory mechanism [6–8].

Based on the existing clone selection algorithm, this paper deeply studies the identification, learning, and defense mechanism of the immune subtype system in hepatocellular carcinoma. The matching mapping relationship between the global optimization problem, the constrained optimization problem, and the dynamic optimization problem, and based on the mapping relationship, the corresponding artificial immune subtype algorithm is proposed to solve the two problems of constrained optimization and dynamic optimization. Based on the dual roles of hepatocytes in innate immune subtypes and adaptive immune subtypes, metaphors were extracted, and the matching mapping of immune subtype responses and constrained optimization problems was constructed. Then, the two forms of candidate solutions caused by the existence of constraints in the constrained optimization problem—feasible solutions and infeasible solutions—are simulated, respectively, with the activation and nonactivation of liver cells. The direction information promotes the infeasible solution to the feasible region and then solves the constrained optimization problem by accurately locating the feasible solution. Short-term memory extracts the important information of the immediate previous environment and plays a role in tracking less severe changes in the external environment, while long-term memory extracts the historical information of the previous environment, which is useful for the cycle of the environment and the design of the initial cells of the cycle-like changes. Experiments verify the effectiveness of the proposed strategy. The IAIS algorithm only uses the traditional artificial immune subtype operator to improve the performance of the algorithm, showing the great potential of the artificial immune subtype optimization algorithm in solving constrained optimization problems.

## 2. Related Work

Evolutionary algorithm is an optimization search method based on the principle of natural selection in the biological world. The evolutionary algorithm simulates the biological evolution process and the operation of fuzzy logic on the computer. It does not need specific knowledge of the object, nor does it need the search space of the object to be continuous and differentiable. It has the ability of global optimization and can solve a problem well. Ontology is used in authority management, and ontology is introduced to conceptually model operation-related information at the business level; and a suitable expression framework for defining and managing generalized operations with business connotations and a wide range is realized. However, it uses traditional database technology to manage and maintain the ontology, which limits the generality and sharability of the ontology itself. In order to improve the shortcomings of the evolutionary algorithm itself, people combine it with some other algorithms to form a new improved algorithm [9–11].

Xue and Sun [12] introduced a new adverse selection algorithm, called the artificial adverse selection evolutionary algorithm, for multilevel classification. It introduces a cutting method that reduces the influence of the Mate parameter. Combining the reverse selection algorithm with the clonal selection mechanism is used to solve the situation that prevents the reverse selection algorithm from being applied to classification problems. These cases include random search, overfitting, and incomplete information. Teo et al. [13] believes that the multiobjective evolutionary algorithm is called the continuous MCDM evolutionary algorithm problem. The main feature of the MODM problem is that the evolutionary algorithm needs to achieve multiple goals, and these multiple goals are conflicting with each other. The MODM model includes evolutionary algorithm variables, objective functions, and constraints. Evolutionary algorithmists try to maximize (or reduce) the objective function, and since there are few unique solutions to this problem, evolutionary algorithmists expect to choose from more efficient solutions (as alternatives). A method (RCMate parameter) for learning fuzzy cognitive graphs from data using real-number evolutionary algorithms is proposed. Bejarbaneh et al. [14] assume that, after the initial state has been determined, a sequence of values for each concept point can be observed on the system to be modeled. The observation sequence is divided into groups of combinations of time *t* and *t* + 1, and the estimated value of time point *t* + 1 can be calculated from the time *t* in each group. The purpose of the learning algorithm is to find the optimal fuzzy cognitive map such that it can produce the same sequence as the system model. This algorithm is used to minimize the error between estimates and observations. Yazid et al. [15] also proposed a scalable divide-and-conquer method based on evolutionary algorithms to learn large-scale fuzzy cognitive graphs. The response sequence is decomposed into several subsequences, and each evolutionary algorithm only focuses on minimizing the output error of one subsequence. Therefore, after all the evolutionary algorithms are executed, several fuzzy cognitive graphs will be generated, and each fuzzy cognitive graph is a weight as the single objective function value. The final fuzzy cognitive map is obtained by calculating the average weight of the subfuzzy cognitive maps.

Valdez et al. [16] introduced an adaptive clone selection (ACS) algorithm, which is a modification of the CLONALG algorithm. The article suggests some modifications to CLONALG based on operator analysis because choosing the number of mutations and clones can overcome the shortcomings of CLONALG, such as using some Mate parameters or representing it in binary. We propose an adaptive immune subtype cloning strategy algorithm (AICSA) to solve numerical optimization problems. According to the affinity of Ab-Ab and Ab-Ag, it dynamically allocates immune subtype memory cells and antibody populations. It also integrates local search and global search [17–19]. The researchers proposed an improved clone selection algorithm based on the CLONALG algorithm. A learning operator is introduced to strengthen the learning mechanism of the CLONALG algorithm and improve the detection efficiency. Scholars have proposed a real-coded clonal selection algorithm (RCSA) for electromagnetic design optimization. It is shown that, with some changes to the clone selection algorithm, the optimization problem of real variables can be solved. It has features such as the number of clones, the mutation range, and the proportion of evolutionary algorithms selected for each generation. Some scholars have introduced an immune subtyping algorithm for continuous global optimization problems, namely OPT-IA. The main feature of the algorithm is that the clone operator explores around each point in the search space. The algorithm is used in the inverse hypermutation operator, where the number of mutations is inversely proportional to the health value. Finally, an aging operator can be used to remove the earliest candidates from existing evolutionary algorithms and introduce diversity [20–25].

## 3. Fuzzy Logic and Evolutionary Algorithm Architecture

### 3.1. Evolutionary Algorithm Test Function

The strategy is to get your own best solution while remembering other fuzzy logic best solutions. The solution to this optimization problem consists of several parameters, each of which is assigned to one of the fuzzy logic. Each fuzzy logic optimizes only its own Mate parameters (its strategy), which act as constants. The rest of the Mate parameter settings are obtained by other fuzzy logic taking the best solution. Solutions from all fuzzy logic should build the solution to the problem. Then, all fuzzy logic uses the immune subtype algorithm to optimize their purpose. In the DMEA algorithm, the authors make full use of the profile information and consider the external profile to be an informative data set, so this profile guides the evolutionary process and improves the quality of understanding through the directional information in it. In this process, the parent individuals are randomly selected, and the offspring are generated by disturbance along the determined improvement direction.

(1) $$\begin{array}{c} \left\{\begin{array}{c} g\left(x,x^{\prime }\right)<f\left(x,x^{\prime }\right),x\leq x^{\prime },\\ \log\;g\left(y,y^{\prime }\right)>\;\log\;f\left(y,y^{\prime }\right),y\leq y^{\prime }. \end{array}\right. \end{array}$$

It can be started from two aspects: on the one hand, the existing knowledge and experience about the genetic algorithm are described in a vague language and used to control the genetic operation and Mate parameter setting online to form a dynamic evolution algorithm; on the other hand, learn from the idea of fuzzy logic and fuzzy set operations and obtain fuzzy codes and corresponding fuzzy genetic operations, in order to achieve the purpose of improving the performance of evolutionary algorithms. By analyzing and establishing the fuzzy mapping relationship between various factors and the optimization ability and convergence speed of Mate parameters, they can be easily integrated together to improve Mate parameters and improve performance. Research shows that in the process of solving the Mate parameter, changing P1 and P-n in a timely and appropriate manner can significantly enhance the optimization ability of the algorithm and greatly improve the convergence speed. Therefore, it can be considered that the basic symbols and their meanings definitely exist in the description logic system, that is, the probability of existence is 1.

(2) $$\begin{array}{c} h\left(u,u+m\left(t\right)\right)-h\left(u+m\left(t\right)\right)=\nabla h\left(m,m\left(t\right)\right)-\frac{\nabla h\left(m,m\left(t\right)\right)}{f\left(m,m\left(t\right)\right)}. \end{array}$$

Each fuzzy logic solution will be attempted to be added to the new cell, and its solution will be added if it can dominate other solutions, and the dominated solution will be removed. Also, if the solution does not dominate any other solution, but it is not dominated, it will also add new cells. The Mate parameter “suppression distance” in the algorithm can prevent solutions from concentrating on a point in space, and solutions smaller than this distance will not be added to new cells. In addition to recognizing antigens, antibodies can also recognize other antibodies. Antibody-to-antibody recognition can be achieved at multiple levels, forming chains of inhibition and enhancement, resulting in complex reactive immune networks that regulate self-matching antibody concentrations. AIS is particularly good at maintaining and promoting diversity. This can be achieved in two ways.

### 3.2. Fuzzy Logic Global Optimization

The theorem shows that, for the set of all possible functions, any optimization search method is equal, that is, no optimization search method is better than other optimization search methods, not even better than a pure random search method. The key to no free lunch theorem is “the set of all possible functions,” which includes both the cheat function and the random function. For these functions, the performance of the function is mostly random. Searching for its optimization is tantamount to looking for a needle in a haystack. It is extremely difficult to find a method with better search performance, and it is not even comparable to a simple random search. However, there is a third class of functions in the set of all possible functions. In general, the distribution of the values of such functions follows a certain law and can provide useful clues for the optimization of the optimal position.

(3) $$\begin{array}{c} P\left(f\times j|f\in S,j\in S\right)=\left\{\begin{array}{c} \frac{f\times j}{\left(f+j\right)\left(f-j\right)},\;j>0,\\ \frac{j}{\left(f+j\right)'\left(f-j\right)'},\;j\leq 0. \end{array}\right. \end{array}$$

This paper adopts the evolutionary algorithm of binary coding. In the iteration of the algorithm, the crossover rate and the mutation rate are not fixed. They are fuzzy changes according to the individual fitness value in the cell as the iterative process progresses, and then the fuzzy control rules are introduced to realize the fuzzification of the evolutionary algorithm, that is, the fuzzy evolutionary algorithm. The basic concept and idea of fuzzy evolutionary algorithm, the detailed design of fuzzy evolutionary algorithm, and its algorithm description and program design are given, and finally the function is used for effective verification. Heterogenesis, on the other hand, involves the introduction of diversity, which can be accomplished through hypermutation of the hepatocyte body or the uptake of new hepatocytes.

A user's multiple interests are realized with an information space that is sufficiently covered by heterogeneity, while also ensuring that it is new and can confirm previously unsatisfied information items (antigens). Heterogenesis further helps to explore new frontiers in the information space. By maintaining and enhancing diversity, it can be shown that these systems effectively adapt to user profiles on the problem of changing short-term and long-term interests of users.

Immune subtype recognition is achieved through the binding of antigen recognition receptors on lymphoid hepatocytes to antigens. The strength of the binding in Table 1 is called affinity. The process of immune subtype recognition is also a self-learning process. The main feature of clonal selection is the clonal proliferation of immune subtype hepatocytes under antigen stimulation, which corresponds to an affinity maturation process, that is, individuals with low antigen affinity undergo proliferation, replication, and mutation operations under the action of the clonal selection mechanism. After that, its affinity gradually increased and is a “mature” process. The immune subtype immune network model regards AIS as an immune network structure composed of lymphoid hepatocytes (antibodies) and achieves immune subtype system functions such as learning, recognition, response, and memory through information transfer and interaction between nodes. Through the relationship between the mutual stimulation and inhibition, the intensity of immune subtype in Figure 1 is ensured and the stable balance of immune subtype response is maintained.

Some of them have higher dimensions, such as the test functions G01, G02, G03, G07, G19, G20, and G22 all have dimensions greater than or equal to 10 dimensions. And some functions have very low feasibility rate, such as G03, G05, G11, G13, G14, G15, G17, G18, G20, G21, G22, and G23; their feasibility rate is less than 0.80%. For these test functions, it is very difficult to find the feasible region of the function due to the low feasibility rate. Under the constraints of equality and inequality constraints, we can see that most of the optimal solutions of multifunctions trigger multiple constraints (except G08, G12, G19), and G22 even triggers 19 constraints. At the same time, it defines a new index to measure the degree of cell diversity and penetrates it into specific genetic operations, so that the selection process can not only obtain better individuals but also increase the diversity of cells.

### 3.3. Evolutionary Algorithm Performance Iteration

Usually defined as the direction from a solution to a better solution, the direction of convergence in multiobjective optimization problems is a non-normalized vector from the dominant solution to the nondominated solution. If the nondominated solution is maintained from a global perspective, the convergence direction is equivalent to the global convergence direction. In the unconstrained multiobjective optimization problem, the dominant solution guided by the convergence direction is easy to find a more suitable position in the evolutionary algorithm space. The divergence direction in a multiobjective optimization problem is a non-normalized vector from a nondominated solution to another nondominated solution.

(4) $$\begin{array}{c} \frac{\left(\sum u+m\left(t\right)-\sum u-m\left(t\right)\right)}{\left(\sum u+m\left(t\right)+\sum u-m\left(t\right)=1\right)}. \end{array}$$

Better propagation inside the cell can be obtained if the solution is perturbed along the divergent direction. Through the analysis of the simulated fuzzy logic signal and the cell fault signal, the superiority of the morphological Mate parameter compared with the traditional Mate parameter analysis and demodulation analysis in eliminating Mate parameters and extracting fault features is demonstrated. Aiming at the insufficiency of CWT gray moment in representing faults under strong background Mate parameters, a gray moment distribution feature extraction method based on MLMW noise reduction is proposed, which greatly improves CWT to describe the characteristics of frequency energy distribution.

It is an adaptive, self-organizing artificial intelligence technology (Figure 2) for solving extreme value problems. The evolutionary algorithm replaces the Mate parameter space of the problem with the coding space, takes the fitness function as the evaluation basis, uses the coding evolutionary algorithm as the evolutionary basis, and establishes an iterative process by implementing the selection and genetic mechanism for the genetic operation of the individual bit string in the evolutionary algorithm. In this iterative process, the important fuzzy logic in the encoded bit string is randomly reorganized, so that the bit string set of the offspring is better than the bit string set of the parent. The evolutionary algorithm simulates the biological evolution process and fuzzy logic operation on the computer. It does not need the specific knowledge of the object, nor does the search space of the object need to be continuous and differentiable, and it has the ability of global optimization. For some problems that are effectively solved by conventional optimization algorithms, more satisfactory results can often be obtained by using evolutionary algorithm optimization techniques.

(5) $$\begin{array}{c} {\sum \left(u+v\left(t\right)\right)}^{2}+\sum_{i=1}^{t}{\left(Y+u-v{\left(t\right)}_{i}\right)}^{2}-\sum v\left(t\right)=0. \end{array}$$

In the evolutionary algorithm, the fitness of each individual increases continuously until a certain limit condition is met. At this time, the individual with the highest fitness value in the evolutionary algorithm is the optimal solution of the Mate parameters to be optimized. It is precisely because of the unique working principle of the genetic algorithm that it can perform a global optimization search in a complex space and has strong robustness; in addition, the evolutionary algorithm basically does not need any restrictive assumptions for the search space (such as continuous, differentiable, single-peak, etc.). The evolutionary algorithm uses random selection as a tool to guide the search process to develop in a more efficient direction by encoding the Mate parameter space. First, the noninferior solution in the neighborhood is selected through the tournament mechanism to initialize the global external file. Then, execute the neighborhood competition operator, and then execute the mutation operator and the crossover operator for each agent with a certain probability and update the file. Finally, a self-learning operator is performed on each agent in the archive, and the archive is updated simultaneously. It is worth noting that the external archives are updated as the entire evolutionary process progresses.

### 3.4. Fuzzy Logic Evaluation Criteria

An evolutionary algorithm is structured if it is based on a well-defined and recurring evolutionary algorithm process. In most cases, structured evolutionary algorithms can be traced back to an algorithm, and evolutionary algorithmists are more or less aware of this, and structured evolutionary algorithms are more suitable for automatic control. More specifically, if the input flow, output flow, and transformation process performed by the system can be clearly described in the three stages information, design, and selection, then a structured evolutionary algorithm can be formulated. In this context, we can also say that each composition stage is structured. An evolutionary algorithm is semistructured when some of its phases are structured and some are unstructured. Most evolutionary algorithms encountered by knowledge workers in public or private enterprises or organizations are semistructured. So, they can leverage the DSS and business intelligence environment in two ways. For the unstructured stages of evolutionary algorithms, intelligent business tools can provide a passive support method that provides timely and flexible access to information.

The side frequency components on the spectrum are the superposition of the side frequency components generated when the two modulations act alone, but since the side frequency components in Table 2 usually have different phases, the superposition should be vector addition, so the sidebands are not symmetrically distributed. In addition, the sideband is usually unstable, the relative phase relationship between the amplitude modulation and the Mate parameter modulation is easily changed by random factors, and the shape of the sideband will also change. These bring great difficulties to cell fault diagnosis. The ideal value of IGD is a number as close to 0 as possible. In order to obtain a better inverse distance, the Pareto solution set needs to cover all parts of the Pareto set. It can be seen from the formula that the closer the results of calculating GD and IGD are to 0, the better the performance of the algorithm. If and only when the convergence and distribution of the Pareto solution set are good, the values of these two indicators are close to 0. Affinity in this case is a scalar index, which contains Pareto dominance and density information. The Pareto intensity is used to measure antibody-antigen affinity.

(6) $$\begin{array}{c} {\sum \max\left(u,u+v\left(t\right)\right)}^{2}+{\sum \min\left(u,u+v\left(t\right)\right)}^{2}={\sum average\left(u,u+v\left(t\right)\right)}^{2}. \end{array}$$

For example, in the intensity Pareto evolution algorithm, the affinity of antibody to antibody is inversely proportional to the sum of the two smallest Euclidean distances between an antibody and the rest of the population. The genetic forgetting operator can be used to simulate the inactivation of certain hepatocytes when an antigen is encountered. Suppress part of the evolved evolutionary algorithm (based on affinity values) and replace with antibodies from memory.

## 4. Construction of Mate Model of Hepatocellular Carcinoma Immune Subtype Based on Fuzzy Logic and Evolutionary Algorithm

### 4.1. Fuzzy Logic Information Transmission Strategy

If only inequality constraints are considered, the line segment EF is constrained, and the shaded area marked in the graph represents the infeasible area of the search space, the original minimum point a becomes the infeasible solution, and only the blank part of the graph is the feasible solution. Then, the global minimum value becomes the original local minimum value C, the equality constraints reduce the search domain in the one-dimensional case. It can be represented by the line segment EF, the feasible region of the entire search space shrinks to only two points *D* and *B*. Compared with the unconstrained condition, the feasible region almost disappears. If the dimension of the function is high, it will be more difficult to find the feasible region. In this example, the global optimum is at point B by comparison. It can be seen from this example that, under the constraints of constraints, the search domain may be reduced, cut off, or even reduced to one or several points, which is particularly difficult to solve for high-dimensional problems.

(7) $$\begin{array}{c} \sum \text{average}\left(0,u,u+v\left(t\right)\right)>\sum \text{average}\left.\left(0,f\left(u+v\left(t\right)\right.\right)\right)>\sum \text{average}\left(0,f\left(u,t\right)\right). \end{array}$$

The larger the evolutionary algorithm scale, the higher the probability of obtaining the optimal solution. However, if the group size is too large, it will inevitably reduce the speed of the evolutionary algorithm. On the other hand, if the proportional selection mechanism is adopted, when the evolutionary algorithm species is very large, a small number of individuals with high fitness will be selected and survive; if it is eliminated, it will affect the formation of the pairing library, thus affecting the crossover operation; while the evolutionary algorithm is too small, it will limit the search space of the evolutionary algorithm and cause the occurrence of premature phenomenon. The evolutionary algorithm of binary code is more commonly used in actual use, and the value range of the number of evolutionary algorithms is generally tens to hundreds. In the case of a single damage point on the rolling elements, the impulse force is generated when the damage point on the rolling elements comes into contact with the outer or inner ring. Since the load density function and path transfer function at the fault point of the rolling element take the cage rotation Mate parameter as the repetition frequency, the modulation Mate parameter of the high-frequency resonance fuzzy logic signal is the cage rotation Mate parameter.

The immune subtype immune network theory believes that, in the absence of antigen stimulation, the body in Figure 3 is in a relatively stable immune subtype state. When the antigen enters the body, this stability is destroyed, resulting in the production of specific antibody molecules. When the antibody molecule accumulates to a certain amount, it will cause an immune subtype response against the idiotype of the immune subtype globulin molecule, that is, the production of anti-idiotype antibodies. However, since the inherent Mate parameter of the rolling element is very high, it is beyond the range of the Mate parameter that can be measured by the general acceleration sensor; compared with the inner ring, the energy required to excite the inherent Mate parameter of the outer ring is much smaller.

(8) $$\begin{array}{c} \left|\left(1-t\right)\left(x\left(s,t-s\right)\right.+\left(1-t\right)\left(y\left(s,t-s\right)\right.+\left(1-t\right)\left(z\left(s,t-s\right)\right)\right|=1,\text{if}\left(i,j\in \text{rand}\left(m,n\right)\right). \end{array}$$

In general, not only the outer ring or the rolling element is damaged, the inherent Mate parameter of the outer ring will be excited, but also when the inner ring fails, the vibration energy will also be transmitted to the outer ring through the rolling element to arouse its inherent Mate parameter. Antibody molecules are also recognized by their anti-idiotype antibody molecules while recognizing the antigen. The production of such anti-idiotypic antibodies plays a crucial role in immune subtype regulation. It inhibits antigen-stimulated proliferating clones and prevents them from proliferating endlessly, thereby maintaining a stable balance of immune subtype responses.

### 4.2. Hepatocyte Multilayer Immune Subtype System

It is widely present in the blood, lymph nodes, spleen, tonsils, and other organs, and its main function is to secrete antibodies and various lymphokines, present antigens, and regulate immune subtypes. Mature hepatocytes reach the non-thymus-dependent regions of peripheral immune subtype organs through blood to settle, and when stimulated by antigens, hepatocytes differentiate and proliferate into plasma hepatocytes and secrete antibodies to implement humoral immune subtype functions. A large number of B cells are produced and die in the body every day, and the stimulation level of hepatocytes depends not only on the stimulation of hepatocyte antibodies by the antigen itself, that is, the degree of binding to the antigen, but also the degree of cooperation with other hepatocytes. If the stimulation level of hepatocytes exceeds a certain threshold, the hepatocytes will split and replicate themselves with a very high Mate parameter and produce mutations in the fuzzy logic. The fuzzy logic code of each hepatocyte is different, and the antibody molecules produced are also diverse. Conversely, if the stimulation level falls below a certain threshold, the hepatocytes stop replicating and die after a period of time.

Assuming that a series of jobs IV are arranged during the operation period of the fuzzy logic signal, the job numbers in Figure 4 are from the starting node 0 to +1, and each job has no priority in the case of R-type resources being limited. Each *f* ∈ *N* job has a definite time *d* and required resources, and such resources are continuously available over the entire fuzzy logic signal range. Nodes 0 and *n* + 1 represent the start and end of the fuzzy logic signal, and the nodes do not take time and certainly do not consume any resources. The time vector *S* is defined as the time to complete the fuzzy logic signal in the case of resource constraints and priority guarantees. The goal of the RAC is then to find a feasible schedule within which the prespecified deadline for the fuzzy logic signal minimizes the total resource cost. The prominent feature of the vibration fuzzy logic signal is the nonstationary time-varying characteristic. Simply using time-domain statistics and FFT methods often cannot fully and accurately locate the fault features and locations. However, the time-frequency domain and time of fuzzy logic signal must be used comprehensively. Only the analysis methods based on the local features of the fuzzy logic signal, such as the scale domain, and incorporating more feature information of the fuzzy logic signal, can accurately judge the fault.

(9) $$\begin{array}{c} \langle \begin{array}{c} \text{for}\left\{i\in x\left(r,t^{i}\right),x\left(r,t^{i-1}\right),x\left(r,t^{i-2}\right),...,x\left(r,t^{1}\right)\right\},\\ between\left\{i\in f\left[t^{i},i\right],\left[t^{i-1},i\right],\left[t^{i-2},i\right],...,\left[t^{1},i\right]\right\}. \end{array} \end{array}$$

In this paper, this indicator is also used to guide the dynamic changes of crossover probability and mutation probability, so that the changes of crossover probability and mutation probability can make self-adaptation according to the relative degree of individual fitness in cells while considering the degree of cell diversity. Finally, through the numerical experiments of typical test functions, and compared with other methods, it is proved that the algorithm has a high convergence rate and fast search speed and is an effective global optimization algorithm. After initial cell generation, antibodies can be cloned for selection. To avoid premature convergence of the active list, a K-means clustering method is introduced to select the best antibodies from the K clusters for diffusion. For the antibody randomly selected in the text, the randomly selected element of each K class is used as the cluster center, the distance between each element and the center position is calculated, the sample is classified into the class where the cluster center is closest to it, and the new cluster center is calculated. The average value of the elements of each cluster formed to get the new center of the cluster, and so on until each cluster does not change.

### 4.3. Evolutionary Algorithm Immune Subtype Mate Operator

Antibodies and antigens are bound by force or chemical bonds. An antibody binds to an antigen, and it is capable of recognizing by pattern complementation matching between its epitope and the epitope of the antigen. The strength of the binding depends on the degree of pattern matching. This binding force is called affinity. Specific antibody molecules have different affinities for different antigens. The average affinity of an antibody molecule can be enhanced by repeated immunization subtypes, a phenomenon known as affinity maturation. Antibodies can also bind to other antibodies because they have both epitopes and idiotypic epitopes. The real number coding method is to represent each fuzzy logic value of an individual with a floating point number in a certain interval (often refers to the real value of the evolutionary algorithm variable), and the coding length of the individual is equal to the number of its evolutionary algorithm variables. The use of floating-point coding can directly perform genetic operations on the phenotype of the solution, which facilitates the introduction of heuristic information related to the problem domain to increase the search ability of the algorithm and improve operational efficiency.

The so-called criteria for evaluating excellent members are generally based on the value of the evaluation function reflected by a hepatocyte or the probability value or fitness occupied in the evolutionary algorithm in Table 3. A liver cell has a larger fitness, then it has more opportunities to enter the next generation of evolutionary algorithms and have more opportunities to develop. Conversely, bad liver cells are not easy to enter into the next generation of computing and may be eliminated. There are various ways to cross, you can start to exchange every element in front of it from the exchange position, or you can only exchange a certain proportion of elements, and so on. The measurement results data of GD and IGD on the standard test function set UF1∼5 show that the DMOAMate parameters have good performance. Moreover, most of the data on the IGD test results show that the performance of the DMOAMate parameter is better than that of the NSMate parameter-II. It can be seen that many satisfactory nondominated solutions are obtained for the DMOAMate parameters, and these nondominated solutions are very close to the Pareto front. Experiments show that all the innovative studies in this paper are effective.

(10) $$\begin{array}{c} \sum_{i,j-i}^{m}\max\left(0,\left|u+mt-i\right|\right)+\sum_{i,j-i}^{m}\max\left(0,\left|mt-i\right|\right)+\sum_{i,j-i}^{m}\max\left(0,\left|u-i\right|\right)=1-f\left(u,i-j\right). \end{array}$$

The defined MUWD combines the morphological filter operator and the multiscale decomposition algorithm, which can adaptively perform nonlinear filtering based on the morphological characteristics of the fuzzy logic signal on several scales, eliminate the Mate parameters on each scale, and decompose the detailed fuzzy logic signal. The morphological opening and closing operations are idempotent, and in order to extract morphological information at different scales during multilayer decomposition, the length of structural elements increases with the increase of the decomposition scale.

In constrained optimization problems, due to the existence of constraints, the feasible region is reduced to small and sometimes disconnected regions, which greatly increases the difficulty of solving the problem. For some equality-constrained problems, the feasible region is reduced to a line, or even a point. Then, for these problems, finding the feasible region itself is already very tricky. Therefore, when dealing with equality constraints, this paper converts equality constraints into inequality constraints by introducing a tolerance threshold *e* and gradually reduces the threshold as the number of iterations increases to restore the conditional requirements of equality constraints.

## 5. Application and Analysis of Hepatocellular Carcinoma Immune Subtype Mate Model Based on Fuzzy Logic and Evolutionary Algorithm

### 5.1. Fuzzy Logic Data Preprocessing

Due to the setting of the heuristic algorithm, the searched cells will be attracted by the extreme points of the function and gradually converge, and the convergence of the population will help the algorithm to locate the extreme points more accurately, but on the other hand, the convergence of the cells will also make it lose diversity, causing premature convergence trapped in local minima. Therefore, in the general design of the algorithm, the cells will always maintain a high diversity at the beginning, explore the entire space, and continue to converge as the search progresses, localizing the extreme points. The balance of algorithm diversity and convergence is always at the core of designing optimization algorithms. For dynamic optimization problems, most of the general heuristic algorithms have already converged when searching for optimization in a static time slice, losing diversity. When the environment changes, it is difficult to restore the global exploration ability in a limited time, which makes dynamic optimization fail.

(11) $$\begin{array}{c} \frac{\sum_{i=1}^{t}Y_{i}\left(1+\text{tim}\left(x\right)\right)+\sum_{i=1}^{t}Y_{i}\left(1+\text{tim}\left(y\right)\right)}{\sum_{i=1}^{t}Y_{i}\left(1+\text{tim}\left(z\right)\right)}⟶\sum_{i=1}^{t}Y_{i}\left(1+\text{tim}\left(x\right)\right)*Y_{i}\left(1-\text{tim}\left(x\right)\right). \end{array}$$

In order to have a satisfactory effect on the dynamic characteristics, the absolute time integral of the error can be used as the minimum *R* scalar function selected by the Mate parameter. The appearance of a penalty function is used, so that the overshoot can be used as one of the optimal indicators. Therefore, the following formula is selected as the optimal index for Mate parameter selection. In the optimization process of the objective function *J*, before the 120th generation, the optimization effect of the fuzzy evolutionary algorithm and the ordinary evolutionary algorithm on the PiDMate parameter is basically the same, and there is almost no major change in them. However, with the increase of algebra, the evolutionary algorithm appears precocious, that is, the optimal fitness value does not change and tends to 24.3933.

(12) $$\begin{array}{c} \left[\begin{array}{c} \begin{array}{c} \sum \partial \left(u+m\left(t\right)\right)\\ \sum \frac{\partial \left(u-m\left(t\right)\right)}{\partial u\left(s\right)} \end{array}\\ \sum \partial \left(u+t\right)\\ \sum \frac{\partial \left(u-m\left(t\right)\right)}{\partial u\left(t\right)} \end{array}\right]-\left[\begin{array}{c} 1\\ \sum \partial \left(u+t\right)\\ 1\\ \sum \partial \left(u-t\right) \end{array}\right]=0. \end{array}$$

Calculate the distance between all records contained in the leaf node, find the two records with the farthest distance and use them as the new semantic center, and follow the remaining center points according to the distance from these two center points. Split the original leaf node into two leaf nodes; judge whether the fuzzy logic signal of the upper node of the leaf node is greater than *L*, if it is greater, the upper node needs to be split with 4; if the number of fuzzy logic signals is less than or equal to *L*, the reading is complete.

The input of the fuzzy controller can be used: the diversity index of the evolutionary algorithm, the maximum and minimum fitness, the current control Mate parameters in Figure 5, and so on. The fuzzy controller should be able to reflect the behavior of the evolutionary algorithm and also be able to see the function of the parameter setting of the evolutionary algorithm and the genetic operator. Since the fuzzy evolutionary algorithm uses the fuzzy controller to optimize the evolutionary algorithm, in order to maintain the EER balance of the algorithm and avoid premature convergence, it is reasonable to use the evolutionary algorithm diversity index to describe the cell convergence.

In this paper, the fuzzy controller of the “look-up table” method is used, so it is necessary to discretize the universe of input and output variables, comprehensively consider the calculation speed and the adjustment accuracy of the Mate parameters, and combine the basic theories of Fc and FA. The domain is discretized as below. In the evolutionary algorithm, the probability of each individual being inherited into the next-generation evolutionary algorithm is determined by the fitness of the individual. Some evolutionary algorithms will converge very quickly, that is, they are easy to fall into local optimum, and some evolutionary algorithms will converge very slowly. Therefore, in the process of running the evolutionary algorithm, the corresponding scale transformation should be carried out on the individual fitness, and the fitness value in an arbitrary distribution state should be planned to a suitable state, so as to improve the competitiveness between individuals and maintain the evolutionary algorithm.

(13) $$\begin{array}{c} \langle \text{z,y,x}\in \text{R}|f\left(x,y\right)=\sum \partial \left(u+t\right)+10\;\sin\left(2\text{pix}+t\right)+10\;\cos\left(2\text{pix}+t\right),\text{if}\left\{\cos\;x>\;\sin\;x\right.. \end{array}$$

First, the agents in the grid use their perception of the environment to exchange information with other agents, cooperate and compete with each other, and use self-learning behavior to conduct in-depth searches. Second, the “average distance” rule is used as part of the tournament selection mechanism to ensure solution diversity during evolution. Finally, two directions are generated at each generation: (1) a convergence direction between a nondominated solution in the outer file and a dominated solution in the cell; and (2) a direction of convergence between two nondominated solutions in the outer file between the solutions. Under the influence of these two directions, the archive information plays a key role in the process of solving multiobjective optimization problems, and it also reflects the nature of mutual cooperation between agents. The reference model gives the expected reference trajectory of the system, the difference between the reference trajectory and the actual output value of the controlled object is used as a variable function of the adaptation value of the evolutionary algorithm, and the antecedents and consequences of the fuzzy control rule are used as the coding Mate parameters of the evolutionary algorithm. The fuzzy control rules are dynamically optimized by the evolutionary algorithm through operations such as replication, crossover, and mutation, so that the fuzzy control rules can be modified online and the control quality of the system can be improved.

### 5.2. Mate Simulation of Hepatocellular Carcinoma Immune Subtypes

Among them, *J* is the fuzzy logic library for constructing immune receptors. By randomly selecting fuzzy logic fragments from these three fuzzy logic libraries in a specific order to form a new complete antibody, this process is called fuzzy logic recombination. In addition, high-frequency mutation is also introduced into the process of antibody production, which is called hypermutation. Fuzzy logic recombination and hypermutation greatly increase the diversity of antibodies and provide the necessary capabilities for dealing with diverse antigens. It interacts in a highly regulated manner, and its biological functions include hepatocyte lytic effects, phagocytosis, and opsonization of microbial and immune subtype complexes, production of inflammation, and clearance and lysis of immune subtype complexes. Only by binding to the antigen, the antibody molecule activates the immune subtype serum complement, assembles the appropriate region of the antibody molecule, and triggers the classical pathway of complement activation until finally a pore-shaped molecular membrane attacks the complex, drilling holes on the surface of the hepatocyte for the external antigen, destroy the external antigen, the antigen is killed, and then further cleared by the complement system.

(14) $$\begin{array}{c} \frac{\exp\left(a\left(z,t\right)+b\left(z,t\right)+c\left(z,t\right)\right)}{\exp\left(a\left(z,t\right)+b\left(z,t\right)\right)}⟶\;\exp\left(a\left(z,t\right)-b\left(z,t\right)\right),z>t. \end{array}$$

For a fuzzy ontology evolution system based on 2-type fuzzy description logic, the basic operations performed on 2-type fuzzy ontology can be divided into the following 16 kinds. The minimum coverage of logical ontology changes, so we call them meta-operations. Other complex operations in the 2-type fuzzy ontology changes, such as merging classes and splitting classes can be combined by combining 2-type fuzzy ontology meta-operations. The biological immune subtype principle is applied to the process of large-scale complex fuzzy logic signal evolution algorithm, and the reasons for the disputes in decision-making information acquisition of large and complex fuzzy logic signals are analyzed. The ability to identify self and non-self extracts the information that evolutionary algorithm users care about from a large amount of information, to distinguish the different interests of evolutionary algorithm users in different users or different time periods, and play the role of information filtering. Drawing on the algorithm of resisting harmful antigens in the process of immune subtyping, the energy error in the artificial immune subtyping system is estimated through immune subtyping calculation, and the solutions with greater risks during operation and maintenance are excluded, and the fuzzy logic of large and complex algorithms is improved. Signals face the complex and difficult mechanisms of evolutionary algorithms.

In the experiment in Figure 6, cells were used as the control object: the liquid level in the container was used as the controlled quantity. The liquid level change in the container is converted into a standard electrical fuzzy logic signal of 4–20 mA and then converted into a digital fuzzy logic signal by the A/D in the I/O interface and sent to the computer and is controlled in the computer according to the set. The algorithm calculates the next control quality from the read liquid level digital fuzzy logic signal and the liquid level set value input input by the keyboard, and converts it into an analog fuzzy logic signal through D/A in the I/O interface. The logic signal drives the opening of the water inlet valve to add water after passing through the power amplifier of the controller, thus realizing the feedback control of the liquid level. The main goal of uniform design is to sample some points from a given point, and these points can be evenly distributed. It is an experimental method that can adapt to multifactor and multilevel experiments. Improve the experimental speed, other experimental design methods are essentially to select representative experimental points within the scope of the experiment, resulting in the search entering a concentrated area without obtaining an excellent solution, but uniform design can achieve the experimental point in the experiment. The range is evenly distributed, which greatly improves the search range.

(15) $$\begin{array}{c} \frac{f\left(h\left(c,t\right)+h\left(c,t-1\right)+h\left(c,t+1\right)\right)-f\left(h\left(c,t\right)+h\left(c,t-1\right)\right)}{\left|\Delta f\left(x,t-1\right)\right|}≙1. \end{array}$$

In the local selection method, each individual is in a constrained environment, called the local neighbor set (in other selection methods, the entire cell is regarded as the neighbor set of the individual), the individual interacts only with its neighbors, and the neighbor set is defined by the cell's distribution structure, and neighbors can be considered as potential mating partners. When selecting, firstly, half of the mating cells uniformly and randomly are selected, then its local neighbors for each selected individual are defined, and mating partners within the neighbors are selected. Therefore, considering the inherent characteristics of the fuzzy logic regulation immune network reconstruction problem, in this chapter, we propose a fuzzy logic regulation immune network reconstruction multiagent evolutionary algorithm based on the fuzzy cognitive graph. In the experimental part, we verified the MAMate parameter FCM-GRN against large-scale artificial data and the DREAM4 standard data set. The experimental results show that the MAMate parameter FCM-GRN can effectively learn the fuzzy cognitive graph of 200 nodes, and the algorithm is able to optimize graphs with up to 40,000 dimension weights. The experimental results show that, even for 10000-dimensional high-dimensional function optimization problems, the multiagent evolutionary algorithm can still achieve good performance, and it is also the first evolutionary algorithm that can handle such high-dimensional functions. The algorithm has also been successfully extended to solve constraint compensation problems and combinatorial optimization problems.

### 5.3. Example Application and Analysis

To test the algorithm, we selected the well-recognized proposed PSPLIB data set, which involves 4 resource types and tested with 30, 60, 90, and 120 activities, respectively. In Shadrokh's article, the J30 data set test of his Mate parameter algorithm is given, and the upper average improvement percentage is calculated from this. Shadrokh sets a random resource unit cost between 1 and 10 for each resource. Although this cost calculation method is not reasonable in this example, the calculation shows the effectiveness of the AIS method. In this paper, the average improvement rate of the cost upper limit of the two algorithms under different 0 conditions and the maximum value of AVI max, AVI max, the minimum value AVI min, the standard deviation SD, and the upper limit average improvement rate are obtained by the formula, in which the highly structured group communication method draws on the basic concept of the Delphi method. The system design takes into account the communication and information requirements framework required by first responders and command and control personnel in the evolutionary algorithm process. In addition, the system also incorporates expert insights and insights from decentralized communities.

After the primary immune subtype response, a certain number of hepatocytes as immune subtype memory hepatocytes remained in the immune subtype system. Thus, the immune subtype system of Figure 7 can quickly react to counter the antigen after encountering antigen A again (secondary response). The secondary response is specific to the antigen responsible for the rapid increase in the number of antibodies in the hepatocyte nucleus of the immune subtype system. It can react rapidly not only to the same antigen but also to antigens with a similar structure to antigen A, a property known as cross-reactivity. The humoral immune subtype response refers to the immune subtype response process in which hepatocytes proliferate and differentiate into plasma hepatocytes and secrete antibodies under antigen stimulation, that is, the humoral immune subtype is an antibody-dominated immune subtype. Hepatocyte immune subtype response refers to the immune response of hepatocyte immune subtype through the cytotoxic effect of toxic hepatocytes and the release of lymphokines from auxiliary hepatocytes.

(16) $$\begin{array}{c} \text{sig}\mathrm{mod}\left(a,b,i\right)=\langle \begin{array}{c} ab+\text{pareto}\left(a,b\right)+\text{pareto}\left(-a,-b\right),a\leq b,\\ ab+\text{random}\left(a,b\right)+\text{random}\left(-a,-b\right),a>b. \end{array} \end{array}$$

The multiobjective optimization algorithm is based on the multiagent evolutionary algorithm, and the direction operator is introduced into the algorithm, the effective information of the nondominated solution set is deeply excavated, and the convergence efficiency of the algorithm is improved. At the same time, the tournament selection mechanism and the “average distance” rule are used to maintain the diversity of the nondominated solution set, so that the nondominated solutions are more evenly distributed on the Pareto front. The verification results of the algorithm on the ZDT data set and the UF data set show that the algorithm has good convergence and diversity. After the cloning and mutation process, new antibodies are generated. Only the best antibodies are kept in the cells. Other elements are eliminated, and the elements remaining in the cell are seeded with new randomly generated solution vectors. In this way, the antibody should have a low completion time, and this mechanism can find the corresponding new search area, take the antibody with higher affinity in the new antibody and insert it into the original cell, and remove the antibody with higher affinity. Using the newly generated cells as the start of a new generation process, cloning and mutation are continued until conditions are met. The first one is instance change, including changes in the class to which the instance belongs and instance additions and deletions; the second change is the change in cluster structure, that is, changes in the clustering results output by the algorithm are caused by changes in data. It can be seen from the above that the incremental hierarchical clustering algorithm will adjust the clustering results when the data set changes, and once the clustering results change, the changes will be recorded corresponding to the execution instructions for generating the changes of the type fuzzy ontology.

Aiming at the lack of self-adaptability of the local features of fuzzy logic signals based on the general method, a feature extraction method based on local waves is studied. A method to improve the feature extraction performance of local wave decomposition is proposed. According to the local wave mutual information in Figure 8, the Mate parameter components and spurious components are eliminated, and the morphological Mate parameter analysis is introduced to suppress modal aliasing and spurious components and improve the performance. The accuracy of fuzzy logic signal decomposition and the timeliness of instantaneous Mate parameter extraction are obtained. On this basis, an information entropy feature analysis method in the local wave domain is proposed to quantitatively describe the complexity of the fuzzy logic signal distribution in the basic mode space. Its effectiveness is verified with an example. The general framework based on the morphological Mate parameters constructs two morphological Mate parameters, the extremum-lifting morphological Mate parameter and the composite structural element morphological nonsampling Mate parameter, which are used to extract the characteristics of the impact fuzzy logic signal. The analysis has a stronger feature extraction ability; the extreme value-lifted shape Mate parameter is applied to the gray moment analysis of the Mate parameter of cells and hepatocytes, and the results show that its ability to describe the local time-frequency energy distribution characteristics of fuzzy logic signals is greatly improved.

## 6. Conclusion

In this paper, a fuzzy cognitive learning algorithm based on multiagent evolutionary algorithm is proposed, and it is applied to the structure reconstruction of fuzzy logic control immune network. The fuzzy cognitive graph is used to model the dynamic control system of the fuzzy logic control immune network. The directed edge with the weight value of [−1, 1] in the graph represents the interaction relationship between the fuzzy logics, the state value in the graph is [0, 1] node represents the activation degree of fuzzy logic, and the multiagent evolutionary algorithm is used to optimize the weight immune network of fuzzy cognitive graph. This algorithm verifies the artificial data of 5 to 200 fuzzy logic nodes and the DREAM4 standard data of 10 to 100 fuzzy logic nodes and compares and analyzes these data with ACO, RCMate parameters, and NHL algorithm. At the same time, the application of distributed computing ideas greatly improves the computing efficiency, making the algorithm suitable for larger-scale complex immune network problems. It shows that the innovative distributed method of this algorithm can well realize the reconstruction of large-scale fuzzy logic regulation immune networks. Aiming at the different importance of features and their correlation and redundancy, combined with local wave analysis, a method to obtain a subset of features beneficial to classification and improve classification performance is studied from two aspects feature extraction and feature selection: kernel principal element analysis. The former maps data to a high-dimensional feature space through kernel principal component analysis and extracts features on the basis of suppressing redundancy and Mate parameters; the latter uses heuristic search strategies to achieve adaptive multifeatures in the process of evolutionary algorithm learning. The effectiveness of the above methods in improving the learning and generalization performance of evolutionary algorithms is verified with examples.

## Figures and Tables

**Figure 1:** Stable balance of immune subtype responses based on evolutionary algorithms.

**Figure 2:** Evolutionary algorithm performance iteration framework.

**Figure 3:** Modulation Mate parameter distribution of fuzzy logic signal.

**Figure 4:** Comparison of local features of fuzzy logic signals.

**Figure 5:** Discrete processing distribution of fuzzy logic data.

**Figure 6:** Topology of hepatocyte immune subtype action.

**Figure 7:** Distribution of immune subtype memory hepatocyte responses based on fuzzy logic.

**Figure 8:** Adaptive distribution of local features of fuzzy logic signals.

**Table 1:** Fuzzy logic configuration file description.

Configuration file	File index	Short-term text	Effective rate error
*H* (*t*, 1)	64	Mutual stimulation	0.058
*H* (*t*, 2)	13	Subtype immune	0.061
*H* (*t*, 3)	39	Lymphoid hepatocytes	0.064
*H* (*t*, 4)	13	Clonal selection	0.067
*H* (*t*, 5)	44	Antigen recognition	0.070
*H* (*t*, 6)	57	Subtype system	0.072
*H* (*t*, 7)	90	Immune network	0.075

**Table 2:** Fuzzy logic evaluation scale.

Logic evaluation	Average value	Covariance value	Mean square error	Mode order
F-01	0.058	0.953	0.295	0.061
F-02	0.061	0.917	0.326	0.064
F-03	0.064	0.881	0.357	0.067
F-04	0.067	0.845	0.388	0.070
F-05	0.070	0.809	0.419	0.072

**Table 3:** Evolutionary algorithm immune subtype process.

Input: when the length of the code string is l	Import numpy as np Import matplotlib.pyplot as plt
Output: operation of the string in the genetic	
Step 1: the strings of a string set	Plt.figure(figsize = (8, 4))
Step 2: illustrate the discussion	Plt.subplot(211)
Step 3: a pattern is a template	Plt.plot(t[:fft_size], xs)
Step 4: describe the schema quantitatively	Plt.xlabel(u“time,” fontproperties = 'fangsong')
Step 5: as the encoding method to	Plt.title(u“500Hz and 50Hz”
Step 6: number of determined positions	Y_*a* = np.array([198,215,245,226,290])
Step 7: that describes a set of strings	Y_*b* = np.array([203,2349,360,368])
Step 8: the binary string is used	Y_*c* = np.array([185,26,200,236,269,216,2])
Step 9: similarities in certain positions	Plt.ylabel(uʺ,fontproperties = “fangsong”)
Step 10: the mode order of mode H	Plt.subplots_adjust(hspace = 0.4)

## Data Availability

The data used to support the findings of this study are available from the corresponding author upon request.
